# Neural Mechanisms With Respect to Different Paradigms and Relevant Regulatory Factors in Empathy for Pain

**DOI:** 10.3389/fnins.2018.00507

**Published:** 2018-07-24

**Authors:** Yien Xiang, Yicun Wang, Shuohui Gao, Xuewen Zhang, Ranji Cui

**Affiliations:** ^1^Jilin Provincial Key Laboratory on Molecular and Chemical Genetic, The Second Hospital Jilin University, Changchun, China; ^2^Department of Gastrointestinal Colorectal Surgery, China-Japan Union Hospital, Jilin University, Changchun, China

**Keywords:** empathy, pain, insula, cingulate cortex, fMRI

## Abstract

Empathy for pain is thought to activate the affective-motivational components of the pain matrix, which includes the anterior insula and middle and anterior cingulate cortices, as indicated by functional magnetic resonance imaging and other methodologies. Activity in this core neural network reflects the affective experience that activates our responses to pain and lays the neural foundation for our understanding of our own emotions and those of others. Furthermore, although picture-based paradigms can activate somatosensory components of directly experienced pain, cue-based paradigms cannot. In addition to this difference, the two paradigms evoke other distinct neuronal responses. Although the automatic “perception-action” model has long been the dominant theory for pain empathy, a “bottom-up, top-down” mechanism seems to be more comprehensive and persuasive. Indeed, a variety of factors can regulate the intensity of empathy for pain through “top-down” processes. In this paper, we integrate and generalize knowledge regarding pain empathy and introduce the findings from recent studies. We also present ideas for future research into the neural mechanisms underlying pain empathy.

## Introduction

Empathy as a multidimensional psychological conception refers to the capacity to share another person’s affect. By observing or imagining the emotional situations of others, we can vicariously experience their affective states in our mind. Empathy enables us to understand people’s feelings when they experience different emotions or sensations such as happiness, sadness, pain, touch, or tickling (Gallese, 2003). de Vignemont and Singer (2006) defined the four essential elements of empathy: (1) an affective state (2) that mirrors (3) and is induced by observing or imagining that of another, (4) and which is accompanied by the awareness of this origin. Pain is another multidimensional psychological experience that integrates somatic sensation, emotion, and cognition. Recently, the overlap of these realms—empathy for pain—has been particularly explored because of its importance and maneuverability in experiments compared with other types of empathy. First, empathy for pain promotes individual perception and understanding of other people’s distress, contributing to prosocial behaviors or altruism to some extent. Second, the perception of someone else’s painful situation might keep individuals vigilant against dangerous stimuli (Jackson et al., 2006b; Decety, 2009). The neural mechanisms that generate empathy for pain have been uncovered through numerous studies using different experimental techniques (Singer et al., 2004; Avenanti et al., 2005; Bufalari et al., 2007; Cheng et al., 2008) and paradigms (Lamm et al., 2011). In this review, we briefly introduce the neural networks of empathy for pain, including common brain areas and those that differ depending on the paradigm. Major theoretical accounts and regulatory factors of the neural responses for pain empathy are also discussed. Finally, we predict the direction of future research for this field.

## Pain Matrix

According to previous studies of pain, a variety of brain regions are activated by painful stimulation, including primary and secondary somatosensory cortices (S1 and S2), cingulate cortex, insula, brain stem, cerebellum, thalamus, amygdala, hippocampus, parietal operculum, and frontal cortex (orbitofrontal, anterolateral, and prefrontal) (Peyron et al., 2000, 2013; Rainville, 2002; Davis and Moayedi, 2013; Duerden and Albanese, 2013; Kucyi et al., 2014; Case et al., 2016; Vachon-Presseau et al., 2016; Walter et al., 2016). This pain-related brain network is generally regarded as the pain matrix. Bradford (Fenton et al., 2015) classified the pain matrix into three different levels. The primary cortical pain matrix comprises S1, S2 (Iannetti and Mouraux, 2010; Fomberstein et al., 2013), parietal operculum, and posterior insula (PI), and is responsible for the perception and location of pain. The secondary cortical pain matrix comprises the anterior insula (AI), anterior cingulate cortex (ACC), hippocampus (Walter et al., 2016) and amygdala, and contributes to the affective experience of pain. The third cortical pain matrix includes the frontal cortex (orbitofrontal, anterolateral, and prefrontal) and medial and posterior cingulate cortex (MCC and PCC), which is proposed to function in imbuing cognitive meaning (**Figure 1**). The first and secondary cortical pain matrix interact to some extent. Some neural connections between the PI and AI have been found, suggesting that the two parts may work together (Ploghaus et al., 1999; Craig, 2002, 2003, 2009; Critchley et al., 2004; Kurth et al., 2010). The third receives and integrates information from the foregoing two and triggers behavioral response. In brief, the somatosensory components of the pain matrix (S1, S2, and PI) are responsible for encoding the location, quality and intensity of nociceptive stimuli (Ploner et al., 1999; Bingel et al., 2003; Maihofner et al., 2006; Bernhardt and Singer, 2012), while the affective-motivational components (AI and ACC) are primarily related to the experience of negative emotions, such as distress or unpleasantness (Kong et al., 2008; Bernhardt and Singer, 2012).

**FIGURE 1:** Three levels of the pain matrix. The primary cortical pain matrix including primary and secondary somatosensory cortices (S1 and S2), parietal operculum, and posterior insula (PI) contributes to pain perception and location. The secondary including the anterior insula (AI), anterior cingulate cortex (ACC), hippocampus and amygdala functions in affect, which is associated with empathy for pain. The third including the frontal cortex and medial and posterior cingulate cortex (MCC and PCC) is associated with cognition.

## Central Brain Areas Governing Empathy for Pain

Almost all relevant functional magnetic resonance imaging (fMRI) experiments have corroborated the fact that pain empathy activates the affective-motivational components of the pain matrix—the AI and MCC/ACC (Jackson et al., 2006b; Singer and Lamm, 2009; Horan et al., 2016; Lerner, 2017; Tomova et al., 2017). Lamm et al. (2011) integrated the outcomes of an image-based meta-analysis of nine separate fMRI pain-empathy studies and a coordinate-based meta-analysis of 32 such studies. The results robustly confirmed that the AI and aMCC/dACC (anterior MCC/dorsal ACC) are the core brain regions related to empathy for pain and support a shared-representations account of pain empathy (pain and empathy for pain share common neural responses) at the neural level. Singer et al. (2004) performed an fMRI study involving 16 couples. An electrode was attached to the back of the male partner’s hand. The female participant was scanned with fMRI while her partner received painful electric stimulation. Bilateral AI, rACC (rostral ACC), cerebellum, and brainstem were activated in both experienced pain and empathic pain. Moreover, the extent of AI and ACC activation was correlated with empathy ratings. Jackson et al. conducted another pain-empathy study using fMRI. Participants were scanned while viewing and evaluating the extent of pain seen in pictures of painful or non-painful hands and feet. The results showed significant activity in several brain regions, including the ACC, AI, cerebellum, and to a lesser extent, the thalamus. Further, activity in the ACC was robustly correlated with the subjective pain ratings (Jackson et al., 2005). These early fMRI studies provided further evidence for the shared-representations account for pain empathy.

However, fMRI alone cannot answer whether the shared-representations model holds true at the neuronal level because of its low resolution in which signals often come from regions that include several different neuronal populations. To provide more credible evidence and to overcome the defects of these kinds of fMRI studies, new methods and techniques are needed. fMRI adaptation (Grill-Spector and Malach, 2001) is one such method that can detect changing responses to long-term exposure to a stimulus. Based on the theory of neuronal fatigue, repeated stimulation of the same population of neurons will induce attenuated responses, whereas responses are not attenuated when a different population is stimulated. This technique can help researchers distinguish whether the responding populations of neurons are the same or different. A study employed this technique to detect the distinct neuronal responses of different races during pain empathy. The participants were asked to watch an adaptor face and a target face consecutively. When the adaptor and the target were of the same race, repetition suppression of event-related potensials in the participant’s brain occurred. When they were of different races, the phenomenon didn’t occur. The results confirmed that the neuronal responses of different races in pain empathy might be different (Sheng et al., 2016). A recent experiment using multivoxel pattern analysis found that seeing one’s hand in pain and experiencing hand pain produced similar fMRI-activity distribution patterns (bilateral AI), by which we can infer that the same neuronal populations are activated for pain and pain empathy (Corradi-Dell’Acqua et al., 2011). In another study, a research group used a placebo analgesia and an opioid antagonist to trigger the reduction and recovery of firsthand pain experiences, respectively. fMRI signals for both empathized pain and experienced pain were subsequently examined. A concomitant reduction of the activities in AI and MCC areas during empathy for pain was observed when the experienced pain was suppressed by the placebo. Likewise, consistent responses also occurred when an opioid antagonist was used. The experiment suggested that empathy for pain might activate some of the same neural components (AI and MCC) as experienced pain (Rutgen et al., 2015a,b). Two double-blind experiments also reached the similar conclusion that the physical painkiller acetaminophen reduces pain empathy (Mischkowski et al., 2016). These findings provide additional insight into the neuronal basis of pain empathy.

As the core neural structures involved in empathy for pain, the AI and MCC/ACC reflect the affective experience that activates our responses to pain and lay the neural foundation for our understanding of our emotions and those of others (Singer et al., 2004). The body’s internal signals are transmitted to the thalamus by afferents, and from the thalamus to sensorimotor cortex and PI. Neurons in the PI then relay the signals to the ipsilateral and contralateral AI. The AI is associated with emotional functions such as pain-related anxiety and anticipatory arousal, while the PI is related to the sensory experience of pain (Ploghaus et al., 1999; Craig, 2002, 2003, 2009; Critchley et al., 2004; Kurth et al., 2010). A conceptual framework implies that the AI might be pivotal for current and future representations of both self- and other-related emotional states, which are crucial for decision-making guidance, adaptive behavior, and homeostatic regulation (Singer et al., 2009). The ACC is important for adjustments in cognitive control (Newman et al., 2015). Medford and Critchley (2010) pointed out that states of global emotional feeling that are brought in by the AI are relayed to the ACC for selection, preparation, and control of appropriate responses. Thus, the combination of the AI and the ACC is responsible for interoceptive awareness and global emotional representations.

Although most papers report that pain empathy triggers neural responses that are similar to those that occur during the direct experience of pain, experienced pain and empathic pain also evoke responses in differing brain regions. First, only direct experienced pain can activate the PI, which is associated with the sensory experience of nociception. In contrast, both experienced pain and empathic pain activate the AI (Ploghaus et al., 1999). Second, while empathic pain merely activates small regions within the cingulate cortex that are related to affective/motivational functions, experienced pain activates a larger portion of the cingulate, including regions associated with motor control (Lamm et al., 2011). Finally, functional connectivity analyses have found that clusters in the periaqueductal gray and midbrain are more connected to the AI during experienced pain, while clusters in dorsal medial prefrontal cortex (dmPFC) exhibit better connectivity to the ACC and AI during empathic pain. These findings indicate that similarly activated regions may be connected to different up/downstream networks (Zaki et al., 2007). These differences may be critical for determining whether an experienced emotion belongs to ourselves or someone else.

## Distinct Brain Areas With Respect to Different Paradigms

It was previously thought that pain empathy only involves affective-motivational aspects of experienced pain, but not the somatosensory elements (Morrison et al., 2004; Singer et al., 2004). However, subsequent studies have overturned that hypothesis by showing that sensorimotor activation also occurs in some situations. Avenanti first recorded pain-related motor responses during pain empathy using transcranial magnetic stimulation (TMS). When the participants watched needles penetrating the target’s hands or feet, the amplitude of motor-evoked potentials were reduced within the corticospinal motor region that corresponded to the muscle that was observed being pierced. Meanwhile, the amount of reduction was correlated with the participant’s subjective ratings of the sensory qualities of the observed pain (Avenanti et al., 2005). Bufalari et al. (2007) found that the amplitude of an event-related potential (ERP) that generally occurs over primary somatosensory cortex (P45) was modulated by seeing a needle pricking the target’s hand. A magnetoencephalography (MEG) study showed an obvious oscillatory suppression in the primary sensory cortex when viewing pictures of painful situations (Cheng et al., 2008). A Japanese research group conducted an fMRI study in which 10 participants were instructed to imagine pain in their own body while viewing pictures of a painful situation. The fMRI results showed a significant activation in secondary somatosensory cortex, along with the AI and ACC (Ogino et al., 2007). Other fMRI studies likely confirmed the existence of somatosensory responses to other people’s pain (Jackson et al., 2006a; Lamm et al., 2007). However, the experiments all used picture-based paradigms in which an explicit location for pain was depicted on a given body part. In contrast, none of the studies that used cue-based paradigms with abstract visual signals found somatosensory components in the responses to empathic pain. Therefore, we propose that whether somatosensory responses occur during pain empathy depends on the type of paradigm used in the research. Activation of sensorimotor cortex can only be triggered when the observer attends to the painful area in a picture and emphasizes the sensory aspect of pain (Lamm et al., 2007, 2011). Note that similar sensory responses are also induced by non-painful control pictures and are always bilateral (Lamm et al., 2011). It seems that sensory activation generated by picture-based paradigms results from rather unspecific activation that is based simply on having a visual stimulus that represents a body part, rather than pain empathy itself (Keysers et al., 2010). Nonetheless, the activation intensity triggered by painful pictures is higher, suggesting that general somatosensory responses elicited when exposed to images of body parts can be amplified by painful situations (Lamm et al., 2011).

The two paradigms generate other distinct neural responses in addition to somatosensory activation (**Figure 2**). Picture-based paradigms always induce activation of the ventral premotor cortex and the anterior inferior parietal cortex. This cortical network is associated with observing, understanding, and imitation of actions (Rizzolatti et al., 2006; Jabbi and Keysers, 2008; Van Overwalle and Baetens, 2009). The recruitment of this network might be related to understanding and predicting the outcome of the situations being viewed, which in turn influences affective state (Schubotz, 2007; Lamm et al., 2011). Cue-based paradigms appear to recruit brain areas related to mentalizing, such as the precuneus, temporo-parietal junction (TPJ), ventral parts of medial prefrontal cortex (mPFC), posterior superior temporal cortex, and temporal poles (Gallagher and Frith, 2003; Van Overwalle and Baetens, 2009). This complicated network is thought to be crucial for sharing in someone else’s emotional state according to one’s own previous knowledge and experience (Schilbach et al., 2008; Laird et al., 2009; Mitchell, 2009).

**FIGURE 2:** Common and distinct brain areas associated with the two paradigms. The common neural network activated in both picture-based and cue-based paradigms is the affective components of the pain matrix including the AI and MCC/ACC. Picture-based paradigms trigger distinct responses in somatosensory regions of pain including S1 and S2, and some brain areas for action observing, understanding and imitation including the ventral premotor cortex and the anterior inferior parietal cortex. While cue-based paradigms uniquely activate regions for mentalizing including the precuneus, temporo-parietal junction (TPJ), ventral parts of medial prefrontal cortex (mPFC), posterior superior temporal cortex, and temporal poles.

## Theoretical Accounts and Regulatory Factors for Neural Responses of Pain Empathy

Inspired by perception-action models of motor behavior and imitation (Prinz, 2010), Preston and de Waal (2002) came up with a similar model, explaining that in empathy “observation or imagination of someone else in a particular emotional state automatically activates a representation of that state in the observer, with its associated autonomic and somatic responses.” Thus, just as we simulate another person’s action to understand their action with our own motor system, we likely simulate another person’s feelings to understand their feelings with our own emotion system (Keysers and Gazzola, 2006). This became a major theory for the neural responses of pain empathy as soon as it was proposed. However, as researchers delved deeper, they found that many factors can influence the empathy for pain process. Therefore, the simple model seemed an inadequate explanation for this psychological phenomenon. Goubert et al. (2005) subsequently proposed another theory that attributes the sense of knowing another person’s painful experience to both top-down and bottom-up processes, which in turn elicit individual affective and behavioral responses. This theory integrates bottom-up automatic feelings with top-down subjective modulation and is more persuasive with respect to the theoretical account of pain empathy. de Vignemont and Singer (2006) presented an early appraisal model and a late appraisal model as a complement to the bottom-up/top-down theory. The two models were set up to decide the time period when regulatory factors affect emotional states, but subsequent studies revealed that different factors might be “inserted” into the affective process at different times.

The bottom-up affective state is regulated by many top-down factors, including cognitive or contextual appraisal (Gu and Han, 2007; Lamm et al., 2007), attention (Gu and Han, 2007), perceived fairness (Singer et al., 2006), affective links between observers and targets, and group membership (Lamm et al., 2011). Here we briefly introduce some recent advances in research. Preis with his colleagues tested the effect of prior pain exposure on AI and aMCC activity during pain empathy. Participants were asked to view pictures of painful (pain pictures) and painless (neutral pictures) situations. Half the participants were exposed to the pain stimulus depicted in the pictures before seeing them, while the other half were only touched gently. Activity in the aMCC and right AI of the participants who experienced the pain before seeing the pictures was lower than that observed in the other participants. At the same time, those exposed to pain also exhibited stronger activation in retrosplenial cortex, mPFC, and dmPFC. They concluded that prior exposure to pain (prior experience) decreases activity in the core neural networks for pain empathy, and increases activity in regions related to perspective taking and memory retrieval, as a top-down regulation mechanism (Preis and Kroener-Herwig, 2012; Preis et al., 2013). One study tested the modulatory effect of responsibility and the sense of agency on empathy for pain. In the first experiment, participants were asked to watch videos showing people exhibiting facial expressions of pain, but their responsibility for that person’s pain differed among three conditions. In Condition One, the observers could only passively watch the target’s facial expression. In Condition Two, they were required to press a button to deliver an electric shock. In Condition Three, they had to choose the shock intensity (among four levels) before delivering it. The unpleasantness ratings and facial electromyographic responses of the observers increased with their responsibility for deciding the shock level and for delivering the target’s pain. The second experiment found that replacing responsibility with sense of agency produced similar results. The two experiments confirmed that responsibility and sense of agency can enhance pain empathy (Lepron et al., 2015). Another study examined social hierarchies—a completely new regulatory factor for pain empathy. In this experiment, a social hierarchy model was established by a skill-related, dot-estimation task in which all the participants were told that they were mediocre. They were then requested to watch superior and inferior people receiving non-painful or painful stimulation and were then scanned by fMRI. As a consequence, participants experienced higher activity in the AI and aMCC when observing inferior-status people receiving painful stimulation. Further, painful stimuli applied to superior-status people were prone to induce attenuated signals in the affective areas for pain. The empathic preference for inferior-status people was concomitant with co-activations of the thalamus and middle frontal gyrus, which are important for emotional processing and cognitive control. These findings thus indicated that empathy for pain is regulated by social hierarchy and biased toward people of lower rank (Feng et al., 2016). The dorsolateral prefrontal cortex (DLPFC) is related to cognitive appraisal and top-down regulation of experienced pain (Rego et al., 2015; Enzi et al., 2016). A sham-controlled study evaluated empathic pain using bilateral transcranial direct current stimulation (tDCS) over the DLPFC. Valence and arousal evaluations were reduced by left-cathodal/right-anodal tDCS, which suggested the unique effect of lateralized DLPFC activation on cognitive appraisal toward pain empathy. Both left-cathodal/right-anodal and left-anodal/right-cathodal tDCS reduced negative emotions and perception of empathic pain, indicating the distinct roles of the DLPFC in affect regulation (Rego et al., 2015). Another research group designed an fMRI experiment to investigate whether in/out-group decisions influence empathy for pain. Thirty participants underwent fMRI scanning after attending to in/out-group members who were depicted receiving painful or non-painful stimulation in a picture-based paradigm. Signals in pain-related and vision-related regions were observed. The result suggested no in-group bias for empathy ratings, whereas distinct activation differences in parts of the cerebellum, right fusiform gyrus, hippocampus, and amygdala were observed between groups, suggesting that these regions may be associated with the modulation of pain empathy (Ruckmann et al., 2015). There is a commonly recognized phenomenon that non-Caucasian patients are more likely to suffer inadequate pain treatment in North America (Weisse et al., 2005; Burgess et al., 2006; Cintron and Morrison, 2006). To explore an appropriate explanation for the disparity, a Canadian group had 50 Canadian medical students (Caucasian 33, First Nations 6, Asian 8, African American 2, Hispanic 1) watch videos of African–American and Caucasian patients showing facial expressions of pain. After that, they were asked to provide a treatment plan and report their feelings for each patient. The observers displayed both pro-Caucasian treatment and empathy bias. Thus, they were likely to present more empathy for Caucasian people’s pain and give them more treatment. The result suggested that racial/ethnic differences might modulate pain empathy (Kaseweter et al., 2012). However, this study was only based on rating scales, and additional research should examine brain activity in these situations. Luo et al. (2014) divided the participants into two groups (one primed with increased mortality salience and the other primed with negative emotion) and scanned them when they were viewing videos of other’s painful situations. They found that the activity of midcingulate cortex could be reduced by reminders of mortality during pain empathy, which is ascribed to the subjective fear of death (Luo et al., 2014). Another study by Luo et al. (2014) found that one’s racial in-group prejudice of neural activity during empathy for pain could be decreased by priming independent self-construals (Wang et al., 2015).

## Future Expectations

Just 20 years ago, empathy for pain was only a psychological conception whose underlying neural mechanisms were almost completely unknown. Recently, with advances in experimental techniques, neuroimaging, and interdisciplinary research, a body of studies have focused on exploring the neural mechanisms of empathy for pain. The underlying neural network has become clearer but is still far from complete. The idea that part of the neural network sub serving empathy for pain is shared with that for experienced pain still remains uncertain and more reliable evidence is needed at the neuronal level using techniques beyond fMRI. Further, the exact reason why picture-based paradigms lead to activation of somatosensory-relate brain regions during pain empathy still needs further discussion. A novel experimental design with modified paradigms might be essential for further investigation. Finally, recent studies on factors that influence empathy for pain are superficial. Corresponding regulatory brain areas and their connectivity with the commonly activated regions during pain empathy need to be discovered. We expect that the neural mechanisms underlying empathy for pain will be completely explained in the near future as experimental design and techniques improve. As above mentioned, empathy for pain can promote individual perception and understanding of other people’s distress and contribute to prosocial behaviors or altruism to some extent, which suggests that empathy for pain might be significant for the treatment of patients with chronic pain, such as those suffering pain by malignancies. Some relevant clinical researches may be focused on this realm.

## Author Contributions

YX contributes to the writing of the paper. YW contributes to the collection of relevant literature. SG, RC, and XZ contributes to the total design and revision of the paper.

## Conflict of Interest Statement

The authors declare that the research was conducted in the absence of any commercial or financial relationships that could be construed as a potential conflict of interest.
